This article has been retracted.

# Leptin Downregulates Aggrecan through the p38-ADAMST Pathway in Human Nucleus Pulposus Cells

**DOI:** 10.1371/journal.pone.0109595

**Published:** 2014-10-09

**Authors:** Zheng Li, Xin Yu, Jinqian Liang, William Ka Kei Wu, Jun Yu, Jianxiong Shen

**Affiliations:** 1 Department of Orthopaedic Surgery, Peking Union Medical College Hospital, Peking Union Medical College, Beijing, China; 2 State Key Laboratory of Cardiovascular Disease, Fuwai Hospital, National Center for Cardiovascular Diseases, Chinese Academy of Medical Sciences and Peking Union Medical College, Xicheng District, Beijing, China; 3 Department of Anaesthesia and Intensive Care, The Chinese University of Hong Kong, Hong Kong; Virgen Macarena University Hospital, School of Medicine, University of Seville, Spain

## Abstract

The mechanistic basis of obesity-associated intervertebral disc degeneration (IDD) is unclear. Aberrant expression of aggrecan and its degrading enzymes ADAMTS-4 and ADAMTS-5 is implicated in the development of IDD. Here, we investigated the effect of leptin, a hormone with increased circulating levels in obesity, on the expression of aggrecan and ADAMTSs in primary human nucleus pulposus (NP) cells. Real-time PCR and Western blots showed that leptin increased the mRNA and protein expression of ADAMTS-4 and ADAMTS-5 and reduced the level of aggrecan in NP cells, accompanied by a prominent induction of p38 phosphorylation. Treatment of NP cells with SB203580 (a p38 inhibitor) abolished the regulation of aggrecan and ADAMTSs by leptin. Knockdown of ADAMTS-4 and ADAMTS-5 by siRNAs also attenuated the degradation of aggrecan in leptin-stimulated NP cells. To conclude, we demonstrated that leptin induces p38 to upregulate ADAMTSs and thereby promoting aggrecan degradation in human NP cells. These results provide a novel mechanistic insight into the molecular pathogenesis of obesity-associated IDD.

## Introduction

Musculoskeletal disorders of the spine are leading causes of disability in people younger than 45 years old and result in national economic losses of more than 90 billion dollars per year in China [1]. Disc degeneration of the spine is considered to be one of the underlying factors of low back pain [2]. Intervertebral disc degeneration (IDD) is a multi-factorial process that is influenced by lifestyles, genetic predisposition, co-morbidities, and aging [3]. The intervertebral disc has a complex structure with the nucleus pulposus (NP) encapsulated by endplates and the annulus fibrosus [4]. The pathogenesis of IDD is poorly understood, although it is known to be associated with a variety of cellular and biochemical changes. One of the most important biochemical hallmarks of IDD is extensive degradation of extracellular matrix (ECM) [5]. The ECM is constantly synthesized and degraded by disc cells in which the rates are normally in balance. However, the balance is shifted towards degradation in IDD, with alterations in collagen type and a decrease in proteoglycan content, leading to the loss of tissue integrity [6]. To this end, the loss of aggrecan, a major type of proteoglycan, is considered to be an early biochemical abnormality of IDD [7].

Aggrecan, a negatively charged proteoglycan, is a major macromolecular component of ECM. The aggrecan monomer consists of a 250 kDa protein core with chondroitin sulfate and keratan sulfate glycosaminoglycan (GAG) side chains attached [8]. Degradation of aggrecan results in dehydration of the disc, which leads to a reduced resistance to compressive load and a reduction in disc height [9]. In the cartilage, two major aggrecanases, a disintegrin and metalloproteinase with thrombospondin motifs 4 (ADAMTS-4) and 5 (ADAMTS-5), are involved in the breakdown of aggrecan [10]. In addition, both ADAMTSs expression are elevated in the NP of human degenerative disc disease [11]. However, the regulation of ADAMTS-4 and ADAMTS-5 expression in NP cells is unknown.

Obesity is a risk factor for IDD, and recent findings indicate that adiposity rather than the excess in body mass is detrimental to the intervertebral disc [12], [13]. The contribution of adiposity-associated metabolic factors to the pathogenesis of intervertebral disc disorders has been the subject of increasing investigations. Leptin, a key cytokine secreted by adipose tissue, has been implicated in many obesity-associated diseases [14]. The serum levels of leptin are about 5 times higher in obese subjects than in normal individuals, with an average of 40 and 8 ng/ml, respectively [15], [16]. The major function of leptin is to mediate signals from the central nervous system to inhibit food intake and stimulate energy expenditure. Accumulating data suggests that leptin could play key roles in many other physiological processes, such as lipid metabolism, hematopoiesis, immune function, angiogenesis, reproduction, bone formation and inflammation [17]. As a mitogenic factor, leptin has been shown to stimulate the proliferation of cancer cells of different tissue origins, including prostate, breast, liver, colon and kidney, via binding to its long isoform leptin receptor (OB-Rb) [18]–[21]. Interestingly, recent studies also indicate that leptin could regulate cell functions in intervertebral disc tissue which expresses functional leptin receptor [22]. To this end, the expression of OB-Rb is upregulated in advanced osteoarthritis and correlated with the body mass index in patients with IDD [12]. Nevertheless, the role of leptin in ECM remodeling, in particular aggrecan degradation, remains unclear.

The aim of the present study is to investigate the effects of leptin on the expression of aggrecan and its degrading enzymes ADAMTS-4 and ADAMTS-5 as well as the associated cellular mechanisms in human NP cells.

## Materials and Methods

### Ethics

All of the experimental protocols were approved by the Clinical Research Ethics Committee of the Peking Union Medical College Hospital. Human lumbar intervertebral disc samples were obtained from patients undergoing discectomy following fully informed written consent of patients.

### Reagents

The p38 mitogen-activated protein kinase (MAPK) inhibitor SB03580 was purchased from Sigma. All primary antibodies and siRNAs were purchased from Santa Cruz Biotechnology.

### Isolation and culture of human NP cells

The human NP cells were dissected from patient underwent surgeries for idiopathic scoliosis (n = 4; average age 20±1.83, range 18–22 years, and Thompson degeneration grade 1). NP cells were isolated and cultured as previously described [12], [13]. After isolation, NP cells were resuspended in DMEM containing 10% (v/v) fetal bovine serum (FBS; GIBCO, NY, USA), 100 µg/ml streptomycin, 100 U/ml penicillin and 1% (w/v) L-glutamine, and then incubated at 37°C in a humidified atmosphere with 95% (v/v) air and 5% (v/v) CO_2_. The confluent cells were detached by trypsinization, seeded into 35-mm tissue culture dishes in complete culture medium (DMEM supplemented with 10% FBS, 100 µg/ml streptomycin and 100 U/ml penicillin) in a 37°C, 5% (v/v) CO_2_ environment. The medium was changed every 2 days. The second passage was used for subsequent experiments.

### Cell transfection

ADAMTS-4 siRNA, ADAMTS-5 siRNA or control siRNA pool was transfected into human NP cells by DharmaFECT1 Reagent (Dharmacon, TX, USA) at a final oligonucleotide concentration of 10 nmol/L according to the manufacturer's instructions. For each cell transfection two or three replication experiments were performed.

### Western blots

Western blots were carried out using standard methods. Proteins were separated on 10% SDS-PAGE, and then transferred to PVDF membranes (Amersham, Buckinghamshire, UK). Membranes were blocked overnight with 5% (w/v) non-fat dried milk and incubated for 2 h with anti-aggrecan antibody, anti-ADAMTS-4 antibody, anti-ADAMTS-5 antibody, anti-p38 antibody or anti-p-p38 antibody at 1∶1000 dilution or anti-GAPDH antibody (Proteintech,Chicago, USA) at 1∶50,000 dilution. After washing with TBST (10 mM Tris, pH 8.0, 150 mM NaCl, and 0.1% Tween20), the membranes were incubated for 2 h with goat anti-rabbit antibody (zsgb-bio, Beijing, China) at 1∶5000 or 1∶50000 dilution (for GAPDH).

### Real-time RT-PCR

Total RNA was extracted from NP cells using TRIzol reagent (Invitrogen, CA, USA) according to the manufacturer's instructions. RNA was isolated with chloroform and isopropanol, washed with ethanol, and dissolved in water. Quantification of RNA was based on spectrophotometric analysis at 260/280 nm with values between 1.8 and 2.0 confirmed the purity of the RNA samples. A 2-µg sample of total RNA was reverse-transcribed with 200 U of MMLV reverse transcriptase (Invitrogen) using Oligo(dT) primers in a 20 µL reaction mixture following the manufactures' instructions. Relative transcript levels of aggrecan, ADAMTS-4 and ADAMTS-5 were determined by real-time PCR using the iQ5 Real-Time PCR Detection System (Bio-Rad, California, USA). The real-time PCR reaction was composed of 1× SYBR Green fluorescent dye (Takara, Dalian, China), 1 µl forward primers (10 µM), 1 µl reverse primers (10 µM), 1× qPCR mix, 1 µl cDNA. The sequences of the specific primers are shown in Table 1. To produce the melting curve, the reactions were subject to one step at 95°C for 30 s followed by 45 cycles of 95°C for 5 s, 60°C for 10 s, and 72°C for 30 s. The relative gene expression was assessed by the ΔΔCt method. GAPDH was used as an internal control.

**Table 1:** Primer sequence.

Name	Sequence (5′-3′)
GAPDH	Forword:TCAACGACCACTTTGTCAAGCTT
	Reverse: GGTGGTCCAGGGGTCTTAC
aggrecan	Forword: CTACCAGTGGATCGGCCTGAA
	Reverse: CGTGCCAGATCATCACCACA
ADAMTS-4	Forword: ACTGGTGGTGGCAGATGACA
	Reverse: TCACTGTTAGCAGGTAGCGCTTT
ADAMTS-5	Forword: GGACCTACCACGAAAGCAGATC
	Reverse: GCCGGGACACACGGAGTAC

### Statistical analysis

Results were expressed as means ± SD of multiple experiments. Statistical analysis was performed with Student's t-test for comparison between two groups. *P* values less than 0.05 were considered statistically significant.

## Results

### Leptin inhibited aggrecan expression

Treating NP cells with leptin (10 ng/ml) significantly reduced aggrecan mRNA levels in a time-dependent manner, with the maximal response at 48 h. Dose-response analysis demonstrated that leptin at the concentration of 1000 ng/ml at the 48 h time point could maximally reduced aggrecan mRNA levels (Fig. 1A). To further investigate whether the reduction in aggrecan mRNA was paralleled by a decrease in aggrecan protein level, Western blot was performed (Fig. 1B). Similar to the effect of leptin on aggrecan mRNA, time-dependent reduction in aggrecan protein expression by leptin was observed.

**Figure 1:** Leptin inhibited aggrecan expression. (**A**) Leptin (10 ng/ml) significantly inhibited aggrecan transcription in a time-dependent manner, with a maximal response both at 48 h. Dose-dependent studies demonstrated a maximal response to leptin (1–1000 ng/ml) was at the concentration of 1000 ng/ml at the 48 h time point. (B) The effect of leptin on aggrecan protein expression was detected with western blotting ananlysis using GAPDH as an internal control. Error bars represent standard deviration.

### Leptin promoted ADAMTS-4 and ADAMTS-5 expression

As shown in Fig. 2, treating NP cells with leptin (10 ng/ml) significantly increased ADAMTS-4 and ADAMTS-5 mRNA levels in a time-dependent manner, with the maximal response both at 48 h. Dose-response analysis revealed that the maximal response to leptin (1–1000 ng/ml) occurred both at the concentration of 100 ng/ml (48 h) (Fig. 2A). Western blot was then performed to further investigate whether the induction of ADAMTS-4 and ADAMTS-5 by leptin occurred at protein level. Results showed that leptin could time-dependently increased ADAMTS-4 and ADAMTS-5 protein expression (Fig. 2B).

**Figure 2:** Leptin promoted ADAMTS-4 and ADAMTS-5 expression. (**A**) The effect of leptin on ADAMTS-4 and ADAMTS-5 mRNA expression assessed using Real-time RT-PCR. For the dose-dependent studies, NP cells were treated with either medium only or varying concentrations of leptin (1–1000 ng/ml) for 24 h. For the time-depent studies, NP cells were treated with either medium only or leptin (10 ng/ml) for varing time intervals (0–72 h). (**B**) The effect of leptin on ADAMTS-4 and ADAMTS-5 protein expression was detected with western blotting ananlysis using GAPDH as an internal control. Error bars represent standard deviration. The medium was changed every day. *p<0.05, ** p<0.01, and ***p<0.001.

### Leptin induced p38 MAPK phosphorylation in human NP cells

Previous studies have shown that p38 MAPK could regulate aggrecan expression in chondrocytes [23]. As shown in Fig. 3A, leptin time-dependently increased p38 phosphorylation of without altering the total protein levels in human NP cells. The stimulation of p38 phosphorylation could be observed as early as 5 min after leptin (10 ng/ml) promotion. These findings indicate that leptin could readily activate p38 MAPK pathways in human NP cells.

**Figure 3:** Pharmacological inhibition of p38 MAPK pathways prevented the regulation of aggrecan, ADAMTS-4 and ADAMTS-5 by leptin. (**A**) The protein amouts of phosphorylated forms of p38 (P- p38 were detected with western blotting analysis. GAPDH was also detected for a loading control. (**B**) NP cells were treated with vehicle (contorl) (-), 10 ng/ml leptin (+), 10 µM SB203580 for 48 h. The amouts of aggrecan, ADAMTS-4 and ADAMTS-5 protein were detected with western blotting analysis using GAPDH as an internal control. (**C**) Aggrecan, ADAMTS-4 and ADAMTS-5 mRNA expression were detected with Real-time RT-PCR analysis using GAPDH as an internal control. Error bars represent standard deviration. The medium was changed every day.***p<0.001.

### Pharmacological inhibition of p38 MAPK pathways prevented the regulation of aggrecan, ADAMTS-4 and ADAMTS-5 by leptin

To examine the possible involvement of p38 MAPK pathway in mediating the effects of leptin on ECM remodeling, NP cells were treated with or without SB203580, in the absence or presence of leptin. Western blot and Real-time RT-PCR analysis show that SB203580 blocked leptin-induced alterations in aggrecan, ADAMTS-4 and ADAMTS-5 protein and mRNA expression (Fig. 3B and 3C).

### ADAMTS-4 and ADAMTS-5 silencing attenuated leptin-induced aggrecan degradation in NP cells

We examined the effect of silencing ADAMTS-4 and ADAMTS-5 expression on aggrecan degradation in human NP cells. ADAMTS-4 and -5 protein levels in the NP cells were significantly reduced by transfection with respective siRNA (Fig. 4A). We then used Western blot to measure aggrecan protein levels in ADAMTS-silenced NP cells. Suppression of ADAMTS-4 and -5 expression significantly restored aggrecan protein expression, indicating the contribution of these two aggrecanases to leptin-induced aggrecan degradation in NP cells (Fig. 4B and 4C).

**Figure 4:** ADAMTS-4 and ADAMTS-5 silencing attenuated leptin-induced aggrecan degradation in NP cells. (**A**) The protein expression of ADAMTS-4 and -5 were detected with western blotting analysis using GAPDH as an internal control. (**B**) NP cells were treated with control SiRNA (SiRNA-con), 10 ng/ml leptin, SiRNA-ADAMTS-4 or SiRNA-ADAMTS-5 for 48 h. The amouts of aggrecan protein were detected with western blotting analysis using GAPDH as an internal control. The signal in each lane was quantified using ImageJ software and the ratio of aggrecan to GAPDH was determined. (**C**) Aggrecan mRNA expression were detected with Real-time RT-PCR analysis using GAPDH as an internal control. Error bars represent standard deviration.

## Discussion

Increasing epidemiological evidence has supported the close association between obesity and IDD [24]. The cellular and molecular mechanism of obesity-related IDD, however, remains unclear. In our study, leptin, a hormone with increased circulating levels in obese patients, has been implicated in the pathogenesis obesity-related IDD [22], [25]. We first demonstrated that leptin directly inhibited aggrecan expression and induced ADAMTS-4 and ADAMTS-5 mRNA and protein expression. These alterations were dependent on p38 activation in NP cells. Importantly, both ADAMTS-4 and -5 were functionally involved in leptin-induced aggrecan degradation in human NP cells. These results indicated that leptin could impair aggrecan expression via induction of ADAMTS-4 and ADAMTS-5 in NP cells and thereby contributing to the pathogenesis of IDD.

The ECM provides both mechanical and biochemical signals to NP cells to regulate their survival, morphology and differentiation. Current evidence implicates the loss of ECM in intervertebral disc during IDD in which the loss of proteoglycans, predominantly aggrecan, is considered as an early indicator of IDD. In this respect, Sobajima *et al.* reported that gene expression of aggrecan was abundant in the non-degenerated, healthy IVD, but its expression steadily declined after annular stab. Although the functional importance of aggrecan secretion has been established, the molecular mechanisms controlling aggrecan turnover in cells of the normal and the degenerated disc are not well understood. Here we found that leptin could enhance aggrecan degradation, which might play a detrimental role in obese-associated IDD.

Aggrecanases are proteinases that cleave a particular glutamyl bond in the interglobular domain of aggrecan, thereby releasing the bulk of the aggrecan molecule from the tissue [26]. Tortorella *et al.* identified the first aggrecanase known as aggrecanase 1 or ADAMTS-4 [27]. Later that year, the same research team identified the second enzyme aggrecanase 2, which is now known as ADAMTS-5 [28]. ADAMTS-4 and -5 play a key role in aggrecan degradation [29]. Emerging studies have demonstrated the importance of both ADAMTS-4 and -5 in the degeneration of intervertebral disc. Demircan *et al.* reported that ADAMTS-4 and -5 expression could be detected in herniated intervertebral disc [30], [31]. Pockert *et al.* also found that the mRNA and protein levels of these two aggrecanases were elevated in degenerated human intervertebral disc samples compared to nondegenerated controls [7]. Previous studies showed that ADAMTS-4 and -5 could be upregulated by inflammatory cytokines, such as tumor necrosis factor (TNF)-α and interleukin (IL)-1β, and such regulation was required for cytokine-dependent aggrecan degradation in human NP cells [10]. In the present study, leptin induced a strong expression ADAMTS-4 and -5 at mRNA and protein levels in NP cells where their knockdown by siRNAs remarkably inhibited leptin-induced aggrecan loss in human NP cells. These data presented here strongly suggest a crucial role for leptin-induced ADAMTS-4 and -5 expressions in the breakdown of aggrecan in NP cells during IDD. However, it is noteworthy that letpin by itself reduced aggrecan mRNA levels whereas ADAMTS-4/5 in theory should contribute to aggrecan proteolysis but not to its regulation at the transcriptional level. Nevertheless, contrary to our expectation, ADAMTS-4/5 knockdown also abrogated the repressive effect of leptin on aggrecan mRNA expression, indicating that ADAMTS-4/5 might be required for mediating the transcription-dependent effects of leptin. This finding is concordant with previous data supporting that ADAMTSs may not only function as extracellular effectors, but also play a role in the modulation of intracellular signaling [32].

Aside from investigating the direct effects of leptin on ADAMTS-4 and -5 expression and aggrecan degradation, we delineated the involvement of p38 MAPK pathway whose roles in leptin signaling and aggrecan degradation have been established in other biological contexts [33], [34]. We found that leptin potently induced p38 phosphorylation in human NP cells. Previous evidences indicated that p38 signaling could control ADAMTS-4 and ADAMTS-5 expression in chondrocytes [35]. To this end, Tian *et al.* reported that TNF-α and IL-1β could modulate ADAMTS-4 and -5 expression through p38 [10]. In line with this previous finding, we also observed that the p38 MAPK inhibitor SB203580 could attenuate aggrecan degradation and ADAMTS-4 and ADAMTS-5 mRNA and protein induction caused by leptin. Importantly, our data suggest that leptin-induced aggrecan downregulation could be contributed by both downregulation of aggrecan mRNA as well as increased degradation through ADAMTSs. In this regard, p38 has also been shown to mediate the downregulation of aggrecan mRNA in chondrocytes treated with IL-1β. However, it must be pointed out that TNF-α and IL-1β are known to change ADAMTS-4/5 expression within a few hours [36] whereas leptin downregulated aggrecan or upreuglated ADAMTS-4/5 only after 12-24 hour in the present study. It raised the possibility that the observed effects may be secondary to leptin signaling. To this end, leptin has been shown to up-regulate the production of pro-inflammatory cytokines, including TNF-α, in macrophages [37]. Whether the upregulation of pro-inflammatory cytokines is required for leptin-induced ADAMTS-4/5 expression and aggrecan degradation, nevertheless, warrants further investigation. In addition to p38 MAPK, our previous data indicated leptin could induce STAT3 signaling in NP cells where pharmacological inhibition of JAK2, the upstream regulator of STAT3, could inhibit leptin-induced cell proliferation [36]. In order to identify more druggable targets for obesity-associated IDD, it would be interesting to delineate if JAK2/STAT3 signaling is also involved in leptin-induced ADAMTS-4/5 upregulation and aggrecan downregulation.

Although *in vitro* data supports that leptin-induced aggrecan downregulation is implicated in obesity-associated IDD, further experiments are needed to differentiate the effect of hyperleptinemia from those arising from other metabolic deregulations in obesity. Determining ADAMTS-4/5 and aggrecan expression in NP cells of obese db/db or ob/ob mice, which are deficient in leptin signaling, would definitely provide a clearer picture. Moreover, it would be valuable to measure ADAMTS-4/5 and aggrecan expression in mice injected with leptin, either acute or long-term, to establish the relationship between hyperleptinemia and ECM imbalance in NP cells *in vivo*. In summary, we provide the first evidence that leptin could induce ADAMTS-4 and -5 expression and thereby promoting aggrecan degradation in human NP cells. Leptin could also directly reduce aggrecan mRNA expression and both actions could be mediated by p38 activation. These data suggest that p38 and ADAMTSs are potential targets for pharmacological intervention in obesity-associated IDD.
